The article "Design, Synthesis and Activity Study of Pyridine Derivatives as Highly Effective and Selective TYK2 Inhibitors" was retracted in 2023. Reasons: unreliable results or conclusions; concerns about the peer review; concerns about the citations.

# Design, Synthesis and Activity Study of Pyridine Derivatives as Highly Effective and Selective TYK2 Inhibitors

**DOI:** 10.1155/2022/6383893

**Published:** 2022-05-09

**Authors:** Chaoying Cheng, Mengguang Zhou, Panpan Zhang, Wenjian Qian, Lei Chen, Guorong Chen

**Affiliations:** ^1^Key Laboratory for Advanced Materials and Joint International Research Laboratory of Precision Chemistry and Molecular Engineering, Feringa Nobel Prize Scientist Joint Research Center, School of Chemistry and Molecular Engineering, Frontiers Center for Materiobiology and Dynamic Chemistry, East China University of Science and Technology, 130 Meilong Road, Shanghai 200237, People's Republic of China, China; ^2^Zhejiang Hisun Pharmaceutical Co, Ltd, Taizhou, 318099 Zhejiang, China

## Abstract

Due to the high homology of the ATP sites of the JAK family, the development of selective inhibitors for a certain JAK isoform is extremely challenging. Our strategy to achieve high selectivity for TYK2 relies on targeting the TYK2 pseudokinase (JH2) domain. Based on the clinical compound BMS-986165, through structure-activity relationship studies, a class of acyl compounds with excellent TYK2 inhibitory activity and selectivity to other subtypes of the JAK family was discovered.

## 1. Introduction

The JAKS kinase family includes JAK1, JAK2, JAK3, and TYK2 isoforms. These 4 family members consist of 1100 amino acids with high homology and can be divided into 7 homology domains (JH): JH1 is highly conserved. The kinase domain has catalytic activity; JH2 is a kinase-like domain, which is unique to JAK kinases from other tyrosine kinases. This domain does not have catalytic activity, but can regulate the activity of JH1 [1–3]. JH3-JH4 is SH2 domain, which can specifically recognize and bind activated tyrosine residues. JH5-JH7 are FERM domains, which are relatively conserved and regulate the binding of JAK to receptors. JAK1, JAK2, and TYK2 are widely present in humans, while JAK3 is only present in hematopoietic tissues such as bone marrow and lymphoid [4, 5].

JAK kinases are involved in the signaling of cytokines and regulate immune responses and can be used as targets for the treatment of autoimmune diseases such as psoriasis and rheumatoid arthritis. At present, tofacitinib developed by Pfizer has been successfully marketed, which can effectively inhibit JAK1, JAK2, and JAK3 for the treatment of rheumatoid arthritis. To date, no selective JAK inhibitors have been marketed [1, 3, 6–8].

Tyrosine kinase 2 (TYK2) is a nonreceptor tyrosine kinase belonging to the Janus kinase family (JAKS). We hope to act on different cellular pathways at this target to minimize potential side effects and maximize the desired pharmacological effects. Selective inhibition of Tyk2 may provide therapeutic benefit in the treatment of various diseases such as psoriasis, systemic lupus erythematosus (SLE), inflammatory bowel disease (IBD), rheumatoid arthritis (RA), cancer, and diabetes [9–13].

The article "Design, Synthesis and Activity Study of Pyridine Derivatives as Highly Effective and Selective TYK2 Inhibitors" was retracted in 2023. Reasons: unreliable results or conclusions; concerns about the peer review; concerns about the citations.

Through the research of BMS, it is found that the activity of TYK2 kinase can be regulated by inhibiting the activity of the JH2 region of TYK2, so as to achieve the purpose of selective inhibition. Its developed BMS-986165 is currently in clinical phase 3 and has achieved excellent clinical results. Although BMS-986165 would have been approved in the near future, the highly potent and selective TYK2 inhibitors were still needed. We chose BMS-986165 as a starting point for medicinal chemistry effort and expected to develop a novel class of TYK2 selective inhibitors [14–16].

## 2. Results and Discussion

First, as shown in Figure 1, we try to optimize the upper segment. After changing the triazole group to H, the compound 1 delivered loss in cellular potency (according to Table 1). However, when the methoxy group was replaced by a trifluoromethoxy group (compound 2), the activity was completely lost; when the amino group was replaced by an S or O atom (compound 3), the activity was completely lost. We therefore believe that the upper segment may be more sensitive to activity.

As shown in Figure 2, we try to optimize the right fragment. After the cyclopropanamide was changed to n-butylhydroxy (compound 4) or carboxyl (compound 5), the activity was completely lost. However, when the cyclopropyl group of cyclopropionamide was replaced with Boc-azetidine (compound 6) or acetyl-azetidine (compound 8), the activity was partially lost; when the amide of cyclopropionamide was reversed (compound 7), the activity was completely lost.

In addition, as shown in Figure 3, we try to optimize the left fragment. After the parent nucleus is replaced with pyridine, the deuterated formamide is changed to nitro (compound 9) or urea group (compound 10), and the activity is greatly lost.

As shown in Figure 4, the activity of the parent pyridazine was changed to pyridine, the deuterated formamide was changed to acetyl (compound 11), and the activity was changed to propionyl (compound 12) and cyclopropionyl (compound 13). The activity can be maintained to a certain extent.

As shown in Figure 5, on the basis of compound 12, the activity of compound 14 was slightly decreased by replacing it with 2,2-difluorocyclopropanamide, and the activity of compound 15 was improved by replacing it with (1R,2r)-2-fluorocyclopropanamide.

We selected compound 12 and compound 15 and compared them horizontally with BMS986165, and found that our compounds 12 and 15 are selective inhibitors of TYK2 and have no problem with safety. Neither CYP nor hERG is inhibited, and in vivo, the kinetic properties are also very good. Compared with the exposure of BMS986165, the exposure is increased by 2-5 times, and there is no problem with LMS in various species. Therefore, we further conducted efficacy experiments for horizontal comparison.

The article "Design, Synthesis and Activity Study of Pyridine Derivatives as Highly Effective and Selective TYK2 Inhibitors" was retracted in 2023. Reasons: unreliable results or conclusions; concerns about the peer review; concerns about the citations.

According to the in vivo PD test in mice of the TYK2 project (Figure 6), at the dose of 10 mg/kg, compound 12 was better than BMS-986165 in inhibition of IFN-*γ* stimulation, and compound 15 was comparable to BMS-986165 in inhibition of IFN-*γ* stimulation.

### 2.1. Chemistry

Compound 12: MS m/z (ESI): 421.2 [M+1].

^1^H NMR (400 MHz, DMSO-*d_6_*) *δ* 11.04 (s, 1H), 10.90 (s, 1H), 8.88 (s, 1H), 8.56 (s, 1H), 8.03 (s, 1H), 7.64 (d, *J* =7.7 Hz, 1H), 7.52 (d, *J* =7.9 Hz, 1H), 7.23-7.28 (m, 1H), 3.95 (s, 3H), 3.71 (s, 3H), 3.12 (q, *J* =7.0 Hz, 2H), 1.98-2.01 (m, 1H), 1.12 (t, *J* =7.0 Hz, 3H), 0.77-0.80 (m, 4H).

Compound 15: MS m/z (ESI): 439.2 [M+1].

^1^H NMR (400 MHz, DMSO-*d_6_*) *δ* 11.06 (s, 1H), 10.95 (s, 1H), 8.89 (s, 1H), 8.56 (s, 1H), 8.02 (s, 1H), 7.66 (d, *J* =7.2 Hz, 1H), 7.54 (d, *J* =7.1 Hz, 1H), 7.25-7.30 (m, 1H), 4.80-4.99 (m, 1H), 3.95 (s, 3H), 3.72 (s, 3H), 3.11-3.14 (m, 2H), 2.19-2.21 (m, 1H), 1.55-1.63 (m, 1H), 1.11-1.24 (m, 4H).

## 3. Summary

In recent years, while JAK inhibitors have achieved great success, their safety has also attracted widespread attention. For example, in 2019, the FDA approved the world's first JAK inhibitor, Pfizer's tofacitinib (Xeljanz, Xeljanz XR). Raise safety warnings: So the pharmaceutical industry is turning its attention to another member of the family, Tyk2. As Figure 7 shows, we optimize compound 12 with better ADME properties and efficacy based on Bristol-Myers Squibb's clinical compound BMS-986165. Therefore, it also has good application prospects and market scale in the future. TYK2 variant exerted highly protective effects on a variety of autoimmune diseases reduced toxicity and the risk of infection, including IBD (UC and CD), multiple sclerosis, ankylosing spondylitis, and psoriasis [17].

## Figures and Tables

**Figure 1:** The SAR of the upper benzene ring.

**Scheme 1:** Synthetic routes of key compounds.

**Figure 2:** SAR of the cyclopropanamide on the right.

**Figure 3:** SAR of the left amide.

**Figure 4:** The deuterated formamide on the left is changed to an acyl group.

**Figure 5:** Modifications based on compound 12.

**Figure 6:** TYK2 project in vivo PD test in mice: IL-12/IL-18 induces changes in serum IFN-*γ* levels in mice.

**Figure 7:** Comparison of compound 12 and BMS clinical compound.

The article "Design, Synthesis and Activity Study of Pyridine Derivatives as Highly Effective and Selective TYK2 Inhibitors" was retracted in 2023. Reasons: unreliable results or conclusions; concerns about the peer review; concerns about the citations.

**Table 1:** The key compound data.

Cpd ID		BMS986165	12	15
Structure				

Biochemical assay IC50 (nM)	TYK2(JH1)	7.5 *μ*M	>10 *μ*M	>16 *μ*M
	JAK1(JH1)	>10 *μ*M	>10 *μ*M	>16 *μ*M
	JAK2(JH1)	>10 *μ*M	>10 *μ*M	>15 *μ*M
	JAK3(JH1)	2.9 *μ*M	>10 *μ*M	>3.4 *μ*M

IC_50_ (nM) cell pSTAT3 (TYK2)		2.8	15.3	12.1

CYP450 inhibition (*μ*M) 1A2/2C9/2C19/2D6/3A4m/3A4t		>30	>30/>30/10.4/>30/>30/>30	>10

hERG (*μ*M)		>30	50	10.6%inhibition@10 *μ*M

PPB (H/R/M)		88.0/83.9/76.8	96.1/88.9/97.2	96.1/NA/94.6

Rat PK 10 mpk, po, DMSO: PEG200		C_max_/AUC/T_1/2_(1360/9570/3.79)	C_max_/AUC/T_1/2_(3560/25400/1.88)	NA

Mouse PK 2%Tween80/0.5%CMC-Na		CL/AUC/t_1/2_ (18.5/885/2.07) 1mpk, iv C_max_/AUC/T_1/2_/F% (2390/9350/1.24/69%)15 mpk, po	CL/AUC/t_1/2_ (11.0/1440/2.8) 1mpk, iv C_max_/AUC/T_1/2_/F% (3870/25000/1.84/112%)15 mpk, po	C_max_/AUC/T_1/2_ (12700/53400/1.81) 15 mpk, po

LMS, H/D/R/M(T_1/2_,min)		NA/478/316/437	1015/164/126/NA	1613/NA/NA/52

Solubility (*μ*M):		PBS (pH 7.4): 4.84 FaSSIF: 94.9	PBS (pH 7.4): 5.6 FaSSIF: 61.4	PBS (pH 7.4): >100 FaSSIF: 52.85

Dose (mg/kg); T_1/2_ (h); CL (mL/min/kg); Cmax (ng/mL); AUC (ng/mL▪h); F (%); iv: intravenous injection; po: peroral administration.

## Data Availability

No data were used to support this study.
